# A Heart Failure Model Established by Pressure Overload Caused by Abdominal Aortic Contraction in Rat

**DOI:** 10.1155/2022/4412228

**Published:** 2022-10-12

**Authors:** Wang Sheng Dai, Yu-Kun Chen, Shi-Hao Lin, Qiang Chen, Hua Cao

**Affiliations:** ^1^College of Clinical Medicine for Obstetrics and Gynecology and Pediatrics, Fujian Medical University, Fuzhou, China; ^2^Fujian Maternity and Child Health Hospital, Fuzhou, China; ^3^Department of Cardiac Surgery, Fujian Branch of Shanghai Children's Medical Center, Fuzhou, China; ^4^Fujian Children's Hospital, Fuzhou, China

## Abstract

Heart failure is a complex clinical syndrome in which ventricular filling or ejection capacity is impaired due to structural or functional diseases of the heart. In order to establish a stable heart failure model, we investigated cardiac parameters in rats with abdominal aortic contraction and normal rats, including the left ventricular posterior wall diameter (LVPWd), the interventricular septum thickness of end-diastolic (IVSd), the left ventricular end-diastolic diameter (LVEDd), the left ventricular ejection fraction (LVEF), and left ventricular fractional shortening (LVFS). Rats were randomly divided into experimental group (*n* = 20) and control group (*n* = 20). The experimental group underwent modified abdominal aortic constriction, while the control group only isolated the abdominal aorta without constriction. The results showed that the survival rate of rats in the experimental group was 85% after one week of operation, while the survival rate of rats in the control group was 100%. Five weeks after operation, the left ventricular posterior wall diameter (LVPWd) and the interventricular septum thickness of end-diastolic (IVSd) in the experimental group were all increased compared with those in the control group, and the differences were statistically significant (*p* < 0.05); the left ventricular end-diastolic diameter (LVEDd) in the experimental group showed an increasing trend compared with the control group, but *p* > 0.05; compared with the control group, the left ventricular ejection fraction (LVEF) and left ventricular fractional shortening (LVFS) in the experimental group showed downward trend, but *p* > 0.05. 10 weeks after operation, the LVPWd, IVSd, and LVEDd of the experimental group were increased compared with the control group, *p* < 0.05, and the LVEF and LVFS of the experimental group were decreased compared with the control group, *p* < 0.05. Compared with the control group, the BNP of the experimental group increased significantly, *p* < 0.05. The heart weight index and left ventricular weight index of rats in the experimental group were significantly higher than those in the control group, *p* < 0.05. HE staining showed that the myocardial cells in the experimental group increased in volume, disordered cell arrangement, widened gaps, increased nuclear hyperchromia, and uneven staining. This paper provides a theoretical basis for the study of heart failure.

## 1. Introduction

Heart failure is a complex clinical syndrome in which ventricular filling or ejection capacity is impaired due to structural or functional diseases of the heart. It has high morbidity and poor prognosis. It is the common outcome in the development of various cardiovascular diseases and an important cause of death in patients with heart disease [1]. Symptoms of heart failure include fatigue, dyspnea, decreased exercise tolerance, and fluid retention [2]. Abdominal aortic coarctation is a congenital heart disease, which is a malformation of blood vessels. It is a congenital developmental abnormality of the aorta between the innominate artery and the first pair of intercostal arteries, resulting in local lumen stenosis and hemodynamic disorders. The main manifestation is high blood pressure. Other manifestations include headache, diplopia, progressive encephalopathy, intracranial hemorrhage, heart failure, and lower extremity weakness. According to incomplete statistics, there are about 13.7 million patients with heart failure in China [3], and up to 40% of the patients die within one year [4]. Heart failure is a common condition in the elderly, affecting about three million people in the United States and about fifteen million people worldwide. The older the age, the higher the prevalence rate, and among the elderly over seventy-five, the prevalence rate is about 10%. Studies have shown that heart failure manifests as progressive cardiomyocyte apoptosis, inflammatory response, interstitial fibrosis, and myocardial structural remodeling [5]. At present, there is no good way to delay and improve the occurrence and development of heart failure, so there are more and more studies on the occurrence, development, and prognosis of heart failure [6, 7].

Animal experiments are scientific studies conducted using animals in the laboratory to gain new knowledge about biology, medicine, etc., or to solve specific problems. Animal experiments are a necessary process before these studies can enter the clinical stage, so it is very important to develop an animal model with key clinical characteristics of human heart failure [8]. Rodent models are commonly used in cardiovascular disease research because of their ease of handling and feeding, short gestation time, and low maintenance costs. Rats are an ideal choice for heart failure models because of their good reproducibility, high stability, low cost, and easy operation [9].

Our study refers to the method of Camacho et al. to prepare a rat model of heart failure by abdominal aortic constriction, and we improve the surgical procedure [10]. Using the splenic vein as an anatomical marker to find the abdominal aorta can quickly find the abdominal aorta. The abdominal aorta was ligated 0.5 cm above the renal artery to reduce its diameter to 0.7 mm. At 10 weeks after operation, the effectiveness of this method was evaluated in terms of echocardiography, cardiac mass index and left ventricular mass index, cardiac pathological staining, and serum brain natriuretic peptide (BNP) to determine the success of heart failure modeling.

## 2. Materials and Methods

### 2.1. Experimental Animal

A total of forty healthy male Sprague-Dawley rats at eight weeks of age were purchased from Wu's Laboratory Animal Company (SPF grade, animal number: SCXK (Jing) 2019-0008) and were adaptively reared in the Medical Laboratory Animal Center of Fujian Medical University for 3 days (clean grade), weighing 250-300 g. They were randomly divided into the operated group (*n* = 20) and the control group (*n* = 20). All rats were fed with standard rat diet, fed, and watered freely at a temperature of 23 ± 2°C and a humidity of 50%-70%. This research was conducted in strict accordance with the recommendations in the Guide for the Care and Use of Laboratory Animals of the National Institutes of Health. The purpose of Laboratory Animal Care and Use is to promote the humane management and use of laboratory animals by providing information on “improving animal welfare, scientific research, and advancing scientific knowledge related to humans and animals.” The guidelines encourage scientists and research institutions to think carefully and rigorously when using laboratory animals, taking into account the possibility of obtaining new knowledge, ethical care, and alternative use of animals in this way. The guide includes information on the assessment and dissemination of scientific, technical, and ethical issues related to animal use and related research testing and educational biological resources. The animal use program was approved by the institutional animal care and use committee of Fujian Medical University.

### 2.2. Animal Surgery

1. Preparation before surgery: rats were fasted for 8 hours before surgery and had free access to water
2. Prepare autoclaved surgical instruments and materials and the recovery cages
3. Keep the laboratory room temperature at 25-30°C, and use a floor-standing surgical lamp to provide light source for the surgical field of vision
4. Anesthetize rats with 2% pentobarbital (50 mg/kg intraperitoneal) [11]. An adequate plane of anesthesia was confirmed by a negative caudal pinch reflex
5. A rat is placed in a supine position on a surgical platform with a heating pad to hold rat's temperature, and its limbs are fixed with adhesive tape. The rat's abdominal surgical area is shaved with a small animal shaver, disinfected with iodophor, and covered with a disposable sterile hole towel
6. A 1.5 cm incision is made along the midline of the rat's abdomen 1 cm below the xiphoid process of the rat with a scalpel. Open the abdominal cavity and elevate the liver with a small gauze. Use two cotton swabs to push aside the gastrointestinal tract (without pulling it out of the rat's abdominal cavity), find the splenic vein and pierce the peritoneum about 0.5 cm above it, and the abdominal aortic pulsation can be seen (as shown in Figure 1). This is where we have improved

(7) The abdominal aorta is isolated and passed 10 cm long 4-0 silk thread below the abdominal aorta at 0.5 cm above the right renal artery
(8) Tie a loose double knot with silk thread, leaving a 3 mm diameter loop, and lay aside a dulled and crooked 22G needle into the loop. Screw up the knot around the abdominal aorta and the needle, then tie another knot (making sure the knot does not loosen), and then immediately remove the needle to constrict the abdominal aorta to a diameter of 0.7 mm. Cut off the overly long sutures
(9) One milliliter of warm normal saline containing 50,000 U of penicillin is injected into the abdominal cavity. The advantages of this are as follows: on the one hand, it can prevent the infection of the rat abdominal cavity; on the other hand, the rat can absorb some of the saline through the peritoneum to replace fluid loss caused by fasting and surgery
(10) Check that there is no gauze residue in the abdominal cavity of the rat, close the rat's abdominal cavity with 6-0 absorbable sutures, and disinfect surgical site. Wait for the rat to wake up from anesthesia and put it into the recovery cage
(11) Rats in the sham group are operated to separate the abdominal aorta and thread, but without constriction. Suture and disinfect the incision, and then put rats into the recovery cages after anesthesia wears off
(12) Postoperative analgesia in rats is very necessary. We add ibuprofen into drinking water (0.2 mg/ml) for analgesic administration
(13) The survival, body weight, mental state, drinking water, diet, coat color, and activity of the rats in the two groups are closely observed and recorded after operation

### 2.3. Echocardiography

Echocardiography was performed at the end of the 5th and 10th week after operation to evaluate the changes in cardiac function of rats. After anesthesia with 2% pentobarbital (50 mg/kg intraperitoneal), the rats were fixed with adhesive tape in a supine position, and the hair on the pectoral and abdominal area of the rats was shaved with a small animal shaver. The ultrasonic diagnostic apparatus was used to examine LVPWd, IVSd, LVEDd, LVEF, and LVFS of the rats at the parasternal left ventricle long-axis section and abdominal aorta long-axis section.

### 2.4. Collection of Rats' Blood Samples and HE Staining

After echocardiography at the end of 10th week, the anesthetic depth was confirmed by testing the tail reflex of rats. All rats were dissected in the middle of the neck to separate the common carotid artery and collect blood. The blood of rats were centrifuged at 3000 rpm for 10 minutes, and the serums were obtained. The serum BNP levels were tested by enzyme-linked immunosorbent assay. These procedures were carried out in the light of the instructions of the kits (ZCIBIO Technology Co., Ltd., Shanghai, China).

After the rats' blood were collected, the hearts were taken out through thoracotomy. The hearts were fully lavaged with precooled normal saline, the tissues surrounding the hearts were cut off, and the liquids on the surface and in the ventricle of the hearts were dried with filter papers. The cardiac mass was weighed, and cardiac mass index (cardiac mass/body weight, mg/g) was computed. The atria and right ventricle of rats were taken out, while the left ventricle and interventricular septum were preserved. Then, the left ventricular mass was weighed, and the left ventricular mass index (left ventricular mass/body weight, mg/g) was computed. The left ventricle free wall of the rats was sliced into small pieces, and a part of the tissues was immediately put into liquid nitrogen for preservation, and the rest of the parts of the tissues were fixed in 4% paraformaldehyde solution.

Then, the fixed tissues were routinely dehydrated and paraffin-embedded, and the thickness of the sections was 4 *μ*m, stained by HE staining. Hematoxylin-eosin staining is abbreviated as HE staining. HE staining is one of the most basic and widely used technical method in the teaching and research of histology and pathology. Yihong is an acidic dye that can dye the eosinophilic structure of tissues to pink so that the morphology of the entire cell tissue is clearly visible. The tissue sectioning method is a very commonly used test method in teaching, scientific research, and pathological examination, and HE staining is the most commonly used staining method in the process of making sections. After neutral gum sealing piece, pictures were taken under a microscope.

### 2.5. Statistical Analysis

SPSS version 25.0 was used for statistical analysis in the study. The quantitative data were expressed as mean ± standard deviation. The comparisons among the different groups were conducted using Student's *t*-test. The value of *p* < 0.05 indicated that the difference was statistically significant.

## 3. Results

### 3.1. Rats' Modeling Success Rate and General Conditions

One rat died on the first day and two rats died on the third day after operation in the operated group, seventeen rats survived, and the survival rate was 85%. All rats in the sham group survived. The rat that died on the 1st day after operation was dissected, and it was found that its cisterna chyli was injured. The two rats that died on the 3rd day after operation showed no obvious abnormality in the autopsy, and they were considered to have died of surgical stress. The rats in the sham group had normal coat color, diet, activity, and body weight. Compared with the sham group, rats in the operated group had fluffy, dry, and lusterless coats; reduced activity; decreased food intake; and slow weight gain. The above performance became more obvious with the increase of modeling time. At the 10th week, the rats in the operated group developed signs of heart failure such as shortness of breath, unresponsiveness to external stimuli, and mild edema.

### 3.2. Echocardiogram Results

As shown in Table 1, in the operated group after five weeks of operation, the LVPWd and IVSd of rats increased, and *p* < 0.05; the LVEDd of rats had a growth trend, but *p* > 0.05; the LVEF and LVFS of rats showed a decreasing trend, but *p* > 0.05. The results meant that rats in the operated group already showed changes in ventricular muscle hypertrophy after five weeks of modeling but did not reach heart failure. Ten weeks after operation, the LVPWd, IVSd, and LVEDd all increased significantly, and *p* < 0.05; the LVEF and LVFS declined significantly, and *p* < 0.05. These results indicated that rats in the surgical group have a tendency to develop heart failure compared to the control group.

B-mode ultrasound of the abdominal aorta demonstrated that the abdominal aorta of rats in the operated group was significantly narrowed, while the abdominal aorta of rats in the sham group was not abnormal, as shown in Figure 2.

### 3.3. Rats' Serum BNP Results

As shown in Table 2, ten weeks after operation, the BNP of rats in the operated group was significantly higher than that in the sham group, *p* < 0.05.

### 3.4. Rats' Cardiac Mass Index and Left Ventricular Mass Index Results

As shown in Table 3, the heart quality index and left ventricular mass index of rats in the surgical group were significantly higher than those in the sham surgery group 10 weeks after surgery (*p* < 0.05).

As shown in Figure 3, the heart volume was enlarged after abdominal aortic constriction operation.

### 3.5. HE Staining of Rats' Hearts

The HE staining results demonstrated that the myocardial cells in the operated group were disordered, the myocardial fiber bundles were wider, the muscle fibers were loose and edema was present, and the gaps were widened. The myocardial cells in the sham group were neatly arranged and dense, as shown in Figure 4.

## 4. Discussion

Chronic heart failure (CHF) is the ultimate destination of most cardiovascular diseases and the leading cause of death [12]. With the development of evidence-based medicine and the deepening of basic research on heart failure, people have a deeper understanding of the pathogenesis, pathophysiological process, and clinical prevention and treatment of heart failure. Among them, a successful establishment of an animal model is the key step to study the treatment of heart failure. Abdominal aorta constriction in rats is an ideal animal model for studying the pathophysiological process, molecular biological mechanism, and cardiovascular pharmacology of pressure overload heart failure by increasing peripheral circulatory resistance [13]. In traditional modeling technique, the abdominal aorta was found through the median incision in the abdomen of rats, and the diameter of the abdominal aorta was narrowed to 0.7 mm, with a mortality rate of 30%-40% in rats [14]. In this study, the surgical procedure was improved on the basis of the traditional modeling technique. After opening the abdominal cavity of the rat, the splenic vein was used as the anatomical marker to find the abdominal aorta, which could quickly and accurately find the abdominal aorta. In addition, it was not necessary to pull the gastrointestinal tract of the rat out of the body, thereby reducing the possibility of intestinal obstruction. After ten weeks of modeling, the rat CHF model was comprehensively evaluated by means of echocardiography, serum BNP, cardiac mass index, left ventricular mass index, and cardiac pathological slices to confirm that the modeling was successful.

At present, commonly used modeling methods in animal models of heart failure include myocardial infarction caused by surgical ligation of the left anterior descending branch of the coronary artery, volume overload caused by arteriovenous shunting, and pressure overload caused by abdominal aorta contraction [15].

Although the degree of heart failure caused by coronary artery ligation is more severe, it needs complex operation and a high level of operative technique. And open-chest operation and mechanical ventilation lead to tall operative mortality [16, 17]. However, abdominal aortic constriction is a relatively simple surgical procedure and has a low mortality rate. Therefore, abdominal aortic constriction is still the preferred modeling method for many basic studies of left ventricular hypertrophy [18].

When abdominal aortic constriction is used, the renal blood flow is significantly reduced after abdominal aortic constriction in rats, which activates the renin-angiotensin-aldosterone system and brings about sodium and water retention in the body, aggravating the degree of heart failure [19]. In addition, when the renal blood flow is reduced, the angiotensin converting enzyme is activated, and the angiotensin I is converted into angiotensin II, which can make the blood vessels contract strongly, aggravate the afterload of the heart, cause ventricular remodeling, and eventually form a vicious cycle [20, 21]. Ventricular remodeling is a compensatory response to increased cardiac load and an important pathophysiological process in the early stage of heart failure [22, 23]. Myocardial hypertrophy due to increased stress load is an important adaptive and compensatory response of cardiomyocytes to increased ventricular wall stress [24, 25], allowing the heart to maintain the body's need for cardiac output for a period of time without clinical symptoms of heart failure. However, ventricular remodeling induced by prolonged pressure overload is one of the independent risk factors for the deterioration of cardiac function and cardiac death [26, 27].

Our modeling method directly leads to increased afterload of cardiac ejection by constricting the abdominal aorta, thus resulting in stable hypertension that is not susceptible to drug effects, which is conducive to the study of various pathological changes from hypertension-induced cardiac hypertrophy to chronic heart failure and has good clinical relevance [28, 29]. Therefore, the improved model of heart failure in rats caused by abdominal aortic contraction is worth generalizing, and this paper provides a theoretical basis for the study of heart failure.

## 5. Conclusion

In this experiment, the use of splenic vein as an anatomical marker can quickly and accurately locate the abdominal aorta of rats so as to carry out abdominal aortic contraction, and the model of chronic heart failure in rats can be successfully established within ten weeks. The model is highly stable, reproducible, and cost-effective, which is an ideal model for the study of chronic heart failure.

## Figures and Tables

**Figure 1:** Surgical diagram.

**Figure 2:** B ultrasound image of abdominal aorta. (a) and (b) represent rats in the operated group, and the black arrow showed the mold narrowing area. (c) and (d) represent rats in the sham group.

**Figure 3:** On the left was the heart of the sham rat, and on the right was the heart of the operated rat.

**Figure 4:** HE staining image of rat heart. (a) represents rats in the operated group. (b) represents rats in the sham group (magnification, ×200).

**Table 1:** Comparison of echocardiographic measurements between the two groups of rats at the end of the 5th and 10th week after operation.

Group	Time	LVPWd (mm)	IVSd (mm)	LVEDd (mm)	LVEF (%)	LVFS (%)
Sham group (*n* = 20)	5th week	1.79 ± 0.11	1.72 ± 0.31	5.05 ± 0.37	89.50 ± 5.38	54.67 ± 4.97
	10th week	1.92 ± 0.17	1.82 ± 0.23	5.34 ± 0.38	87.82 ± 3.04	52.71 ± 6.81

Operated group (*n* = 17)	5th week	2.40 ± 0.29^∗^	2.21 ± 0.34^∗^	5.22 ± 0.15^#^	86.96 ± 3.89^#^	52.13 ± 3.47^#^
	10th week	2.58 ± 0.50^∗^	2.28 ± 0.40^∗^	6.94 ± 0.65^∗^	59.71 ± 5.41^∗^	30.87 ± 5.21^∗^

^∗^: *p* < 0.05 compared with the sham group. #: *p* > 0.05 compared with the sham group.

**Table 2:** Comparison of BNP between the two groups of rats at the end of the 10th week after operation.

Item	The sham group (*n* = 20)	The operated group (*n* = 17)	*p* value
BNP	73.21 ± 23.48	764.19 ± 221.16	0.001

**Table 3:** Comparison of the cardiac mass index and left ventricular mass index between the two groups of rats 10 weeks after operation.

Item	The sham group (*n* = 20)	The operated group (*n* = 17)	*p* value
Cardiac mass index	2.72 ± 0.42	3.93 ± 0.91	0.001
Left ventricular mass index	2.29 ± 0.49	3.46 ± 0.28	0.001

## Data Availability

The data sets used and/or analyzed during the current study are available from the first author or the corresponding author on reasonable request.

## Abbreviations

CHF: Chronic heart failure
LVPWd: Left ventricular posterior wall diameter
IVSd: Interventricular septum thickness of end-diastolic
LVEDd: Left ventricular end-diastolic diameter
LVEF: Left ventricular ejection fraction
LVFS: Left ventricular fractional shortening
BNP: B-type brain natriuretic peptide.
